# Role of Hepatitis C Virus Induced Osteopontin in Epithelial to Mesenchymal Transition, Migration and Invasion of Hepatocytes

**DOI:** 10.1371/journal.pone.0087464

**Published:** 2014-01-31

**Authors:** Jawed Iqbal, Steven McRae, Thi Mai, Krishna Banaudha, Mehuli Sarkar-Dutta, Gulam Waris

**Affiliations:** 1 Department of Microbiology and Immunology, H. M. Bligh Cancer Research Laboratories, Rosalind Franklin University of Medicine and Science, Chicago Medical School, North Chicago, Illinois, United States of America; 2 Department of Biochemistry and Molecular Biology, The George Washington University, Washington, DC, United States of America; Rutgers, The State University of New Jersey, United States of America

## Abstract

Osteopontin (OPN) is a secreted phosphoprotein which has been linked to tumor progression and metastasis in a variety of cancers including hepatocellular carcinoma (HCC). Previous studies have shown that OPN is upregulated during liver injury and inflammation. However, the role of OPN in hepatitis C virus (HCV)-induced liver disease pathogenesis is not known. In this study, we determined the induction of OPN, and then investigated the effect of secreted forms of OPN in epithelial to mesenchymal transition (EMT), migration and invasion of hepatocytes. We show the induction of OPN mRNA and protein expression by HCV-infection. Our results also demonstrate the processing of precursor OPN (75 kDa) into 55 kDa, 42 kDa and 36 kDa forms of OPN in HCV-infected cells. Furthermore, we show the binding of secreted OPN to integrin αVβ3 and CD44 at the cell surface, leading to the activation of downstream cellular kinases such as focal adhesion kinase (FAK), Src, and Akt. Importantly, our results show the reduced expression of epithelial marker (E-cadherin) and induction of mesenchymal marker (N-cadherin) in HCV-infected cells. We also show the migration and invasion of HCV-infected cells using wound healing assay and matrigel coated Boyden chamber. In addition, we demonstrate the activation of above EMT markers, and the critical players involved in OPN-mediated cell signaling cascade using primary human hepatocytes infected with Japanese fulminant hepatitis (JFH)-1 HCV. Taken together, these studies suggest a potential role of OPN in inducing chronic liver disease and HCC associated with chronic HCV infection.

## Introduction

HCV infection is the leading cause of chronic hepatitis which often results in liver fibrosis, cirrhosis and HCC [1]. HCV genome is a 9.6 kb positive sense single-stranded RNA molecule containing a 5′ untranslated region (UTR), a single open reading frame, and a 3′ UTR [2]. The 5′ UTR contains an internal ribosome entry site (IRES), which regulates cap-independent translation of a polyprotein precursor of ∼3000 amino acids that is cleaved by viral and host cell signal peptidases into structural proteins (core, E1, E2) and nonstructural proteins (p7, NS2, NS3, NS4A, NS4B, NS5A and NS5B) [2]. The molecular mechanisms of HCV replication and pathogenesis have been hampered by the lack of an efficient cell culture system or a suitable small animal model. The development of a productive JFH-1-HCV (genotype 2a) infection system provided a major breakthrough that allows the production of infectious virions in cell culture [3], [4].

HCC is a highly aggressive carcinoma of the liver, and is the third most common cause of cancer related death worldwide. Cirrhosis of any etiology is the most common risk factor for HCC development. Over 90% of HCCs develop in a cirrhotic liver resulting from chronic hepatitis B virus (HBV) or HCV infections, alcoholic cirrhosis, or nonalcoholic steatohepatitis [5]. HCC is a complex and heterogeneous tumor with frequent intrahepatic spread and extrahepatic metastasis [6]. The rate of HCC development among HCV-infected persons ranges from 1% to 4%. As with most solid malignant tumors, hepatocarcinogenesis is considered to be a multistep process involving uncontrolled cellular growth, detachment from the extracellular matrix and invasion into the surrounding tissue, along with modulation of both the immune system and the blood supply to promote tumor growth [7]–[9]. Identifying the primary contributors to the metastatic cascade, especially at the early stages of cellular invasion, may present opportunities for reducing the severity of HCC through new therapeutic intervention.

Previously, HCV proteins (core, NS3, NS5A and NS5B) have been shown to possess oncogenic potential [10]–[12]. Apart from HCV core protein, the role of other HCV proteins in the development of HCC is less clear. HCV core protein is considered a major risk factor for the progression of HCC. The expression of HCV core protein in a transgenic mouse model was found to induce tumor formation in liver [13]. However, the underlying mechanism of HCV-induced HCC remains largely unknown. Studies have also shown that HCV core protein expression either in cell culture or in transgenic mice led to the development of hepatic steatosis, a risk factor that contributes to hepatocarcinogenesis [14]. Oxidative stress and steatosis is supposed to play a pivotal role in the development of liver injury or HCC in chronic HCV infection [15], [16]. Our previous studies have shown the induction of oxidative stress in human hepatoma cells expressing HCV proteins or infected with HCV [17], [18].

OPN is a secreted multifunctional phosphoglycoprotein expressed at high levels in tumors and the surrounding stroma of numerous cancers, including HCC [19]–[22]. Several studies have shown the upregulation of OPN in tumorigenesis, angiogenesis and in response to inflammation and liver injury [19], [20], [23]. Studies utilizing high throughput gene profiling arrays have identified OPN as a target for use as a serum biomarker in predicting tumor metastasis [24]. OPN plays an important role in the progression of chronic liver diseases. Recent studies have shown the correlation of serum OPN level with hepatic inflammation and fibrosis in association with alcohol intake [25]. Previously, several viruses such as murine polyoma virus middle T antigen, HBV X protein, and human immunodeficiency virus (HIV) have been shown to induce OPN which can lead to wound healing, cell migration, invasion and metastasis [26]–[28]. Recently, we have shown that HCV activates OPN via Ca^2+^ signaling and elevation of ROS [29].

OPN is a soluble cytokine and a matrix-bound protein that can remain intracellular or is secreted, hence allowing autocrine and paracrine signaling [30], [31]. Osteopontin mediates biological function through signal transduction by binding to the cell surface receptors such as integrin αVβ3 and CD44 [19]. OPN interaction with integrins αVβ1, αVβ3, αVβ5, α4β1, α5β1, α8β1 transduces cell-matrix signaling directed to increased motility, invasion, and angiogenesis [19], [23], [32]. The arginine-glycine-aspartic acid (RGD) domain of OPN interacts with αVβ3 and induces cell signaling required for cell migration and invasion [19], [23].

In this study, we determined the induction and secretion of OPN, and then investigated the role of HCV-induced OPN in EMT, hepatoma cell migration and invasion. Our studies also demonstrate that HCV-induced OPN interacts with integrin αVβ3 as well as CD44 at the cell surface and induces signaling cascade through phosphorylation/activation of FAK, Akt and Src. Furthermore, our results also show the phosphorylation/activation of these proteins in primary human hepatocytes infected with HCV. Collectively, these observations provide novel insight into the role of OPN activation and secretion in EMT, migration and invasion of human hepatocytes associated with chronic HCV infection.

## Materials and Methods

### Expression Plasmids, Reagents, and Antibodies

The infectious J6/JFH-1 cDNA (genotype 2a) along with the replication-defective JFH-1/GND construct was obtained from Dr. C. Rice (Rockefeller University, NY).

All the antibodies were used according to the manufacturer’s protocols; HCV NS3, NS5A (Virogen, Watertown, MA), actin (Sigma, St. Louis, MO), OPN (R & D Systems, Inc., Minneapolis, MN), p-Akt, p-Src, integrin β3, β6, E-cadherin, N-cadherin, pan-cadherin and PDI (Cell Signaling Technology, Danvers, MA), anti-serum albumin (Thermo Scientific Inc. Rockford, IL), anti-FAK (focal adhesion kinase) (BD Biosciences, San Jose, CA), and anti-CD44 (anti-HCAM) (Santa Cruz Biotechnology, Dallas, TX).

### Cell Lines

The human hepatoma cell line Huh7.5 [33], and human hepatoblastoma cell line HepG2 [34] were obtained from Dr. C. Rice, Rockefeller University, NY, and Dr. A. Mclachlan, University of Chicago, IL, respectively. These cells were grown in Dulbecco’s modified Eagle’ medium (DMEM) supplemented with 10% fetal calf serum, 100 U of penicillin/ml and 100 µg streptomycin sulfate/ml. The cells were incubated at 37°C in 5% CO_2_ incubator. Study of HCV mediated liver disease progression is complicated due to the lack of a convenient small animal model susceptible to virus infection. Cell culture system using human hepatoma cell line, Huh-7/Huh7.5 is widely used in HCV field to study the HCV-mediated liver disease pathogenesis.

### HCV Cell Culture Infection System

The plasmid pFL-J6/JFH1 encoding the HCV J6/JFH-1 genome was linearized with *Xba*I for in vitro transcription using the Ampliscribe T_7_ transcription kit (Epicentre Technologies, WI). Fifteen micrograms of J6/JFH-1 RNA/10 cm plate was delivered into Huh-7.5 cells by electroporation as described previously [4], [35]. Cells were passaged every 3–5 days; the presence of HCV in these cells and the corresponding supernatants were determined as described previously [4]. The cell-free virus was propagated in Huh7.5 cell culture as described previously [4]. The expressions of HCV protein in HCV-infected cells were analyzed using western blot assays. The HCV cell culture supernatant was collected at appropriate time points and was used to infect naïve Huh7.5 cells at multiplicity of infection (moi) of 1 for 5–6 h at 37°C and 5% CO_2_ [4], [35]. The viral titer in cell culture supernatant was expressed as focus forming unit (ffu) ml^-1^, which was determined by the average number of HCV-NS5A-positive foci detected at the highest dilutions as described previously [4]. The cell culture supernatant collected from Huh7.5 cells expressing JFH-1/GND (replication defective virus) were used as a negative control. In most of the experiments, HCV-infected cells were serum starved for 4 h before harvesting.

### Hepatocytes Co-culture System

The primary human hepatocytes were obtained from Dr. Ajit Kumar (The George Washington University, Washington, DC). Briefly, the hepatic stellate cell line (CFSC-8B) [36], were used as a feeder cell layer, and freshly isolated human hepatocytes suspension (Cambrex, Walkersville, MD) was seeded over the feeder cell line in a hepatocyte-defined medium (HDM) as described previously [37]. Primary hepatocyte cultures form spherical masses after 30 days in co-culture. The hepatocyte cultures containing spherical masses were harvested with 0.05% trypsin in HDM (supplemented with 1% FBS) and reseeded in six-well plates and propagated in HDM. The *in vitro* transcribed J6/JFH-1 plasmid was transfected into primary human hepatocytes (PHH) as describe earlier [37]. To determine if HCV particles were released in culture supernatant of transfected PHH, conditioned media was collected and used to infect naïve PHH as describe previously [37]. Total cellular RNA was extracted using TRIzol (Invitrogen, CA), and HCV replication levels were analyzed using QRT-PCR (data not shown). For further studies, PHH or PHH infected with J6/JFH-1 HCV at multiplicity of infection (moi) of 1, were harvested at day 8 postinfection, cellular lysates were prepared by incubating in radioimmune precipitation (RIPA) buffer (50 mM Tris, pH 7.5, 150 mM NaCl, 1% NP-40, 0.5% sodium deoxycholate, 0.1% SDS, 1 mM sodium orthovanadate, 1 mM sodium formate, 10 µl/ml protease inhibitor cocktail (Thermo Scientific, IL) for 30 min on ice.

### Western Blotting and Immunoprecipitation

Mock (Huh7.5), and HCV-infected cells were harvested and cellular lysates were prepared by incubating in RIPA buffer for 30 min on ice. Cell culture supernatants from mock and HCV-infected cells were concentrated (20 fold) using centrifugal filter units (Millipore, MA). Equal amounts of protein from lysates or supernatants were subjected to SDS-PAGE. Gels were electroblotted onto nitrocellulose membrane (Thermo Scientific, IL) in 25 mM Tris, 192 mM glycine and 20% methanol. Membranes were incubated for 1 h in blocking buffer [(20 mM Tris-HCl, pH 7.5, 150 mM NaCl, 0.1% Tween-20, 5% dry milk], probed with primary antibody for 1 h at room temperature (RT) and washed twice for 5 min with blocking buffer without milk followed by incubation with secondary antibody for 1 h at RT. After an additional washing step with blocking buffer, immunoblots were visualized using the Odyssey Infrared Imaging System (Li-Cor Biosciences, Lincoln, NE).

For immunodepletion experiments, cell culture supernatants collected from HCV-infected cells were immunoprecipitated using anti-OPN (10 µg/ml) overnight at 4°C. The immune complexes were incubated with protein G-Sepharose (GE Healthcare, Piscataway, NJ) for 1 h at 4°C to remove OPN through centrifugation. The OPN free supernatants were placed on HepG2 cells.

### Laser-scanning Confocal Microscopy

Mock and HCV-infected cells on coverslip were washed with PBS, fixed with 4% paraformaldehyde for 10 min at RT, permeabilized for 5 min with 0.2% Triton X-100, and blocked for 45 min with 5% bovine serum albumin in PBS. The cells were next incubated with primary antibody against the specific protein for 1 h at RT or overnight at 4°C, followed by incubation with Alexa fluor-labelled secondary antibody (Molecular Probes) for 1 h. After washing with PBS, cells were mounted with anti-fade reagent containing DAPI (4, 6-diamidino-2 phenylindole) (Invitrogen, CA) and observed under a laser scanning confocal microscope (Zeiss LSM 510).

### RNA Interference

HCV-infected cells were transfected with GFP siRNA (siGFP), siOPN, siβ3, and siCD44 according to the manufacturer’s protocols (Santa Cruz Biotechnology). Each siRNA consists of pools of three to five target-specific 19–25 nt siRNA designed to knockdown the target gene expression. For siGFP, siOPN, siCD44 and siβ3 transfections, two solutions were prepared. Solution A: 60 pmols of siRNA duplex was mixed with 100 µl siRNA transfection medium. Solution B: 8 µl of transfection reagent was added to 100 µl siRNA transfection medium. Solution A and B were allowed to incubate at RT for 20 min. After 20 min, solution A and B were combined, and incubated for 20 min at RT. The combined solutions were then added to the cells, and incubated for 5–7 h at 37°C and 5% CO_2_, and the transfection solution was replaced with 2 ml of complete DMEM growth media.

### SYBR Green PCR

Total cellular RNA was extracted from mock and HCV-infected cells using TRIzol (Invitrogen, CA) and DNase treated with RQ1 RNase-free DNase prior to cDNA synthesis. The cDNA was reverse-transcribed from 1 µg of total RNA using reverse transcription kit (Applied Biosystems, CA). Quantitative RT-PCR was carried out using SYBR green master mix (Applied Biosystems) and specific primers. OPN, sense primer-5′- CGAGGAGTTGAATG GTGCATAC-3′; antisense primer-5′-TTTCAGCACTCTGGTCATCCA-3′. 18S rRNA was used as an internal control. 18S rRNA, sense primer 5′-ACATCCAAGGAAGGCAGCAG-3′; antisense primer 5′-TCGTCACTACCTCCCCGG-3′. Amplification reactions were performed under the following conditions: 2 min at 50°C, 10 min at 95°C, 40 cycles for 10 s at 95°C, and 1 min at 60°C. Relative transcript levels were calculated using ΔΔCt method as specified by the manufacturer.

### Northern Blot

Total RNA was extracted from mock and HCV-infected cells as described above. Equal amounts (20 µg) of RNA was loaded onto 1% formaldehyde agarose gels and electroblotted onto nitrocellulose membrane. The membrane was hybridized with 5′- biotinylated OPN DNA probe (5′-CTACTCGTTTCATAACTGTCCTTCCCACGGCTGTCCCAATCAGAAGGCGCGTTCA GGTCCTGGGCAACG-3′) and 28S rRNA (5′-GTAGGTAGGGACAGTGGGAATCTCGTTC ATCCATTCATGCGCGTCACTAATTAGATGACGAGGCATTTGGCTACCTTAAGAGAGT CATAG-3′) overnight at 42°C. The membrane was washed with saline-sodium citrate (SSC) buffer containing 0.1% SDS, followed by incubation with streptavidin (1∶10,000) (LI-COR) and developed by LI-COR, Odessey (Nebraska, USA). The above probes were synthesized from Integrated DNA technology, Coralville, Iowa USA.

### Wound Healing Assays

Mock and HCV-infected cells were plated in 6-well culture plates and grown to approximately 80% confluency before scratching with sterile plastic pipette tip across the monolayer. Cell debris was removed by washing with PBS, and the cells were cultured in serum free media. Images were captured after wounding at 0 h and 48 h post wounding. The percent migration distance was calculated according to the formula: percent migration distance = percent initial wound width at time zero – percent wound width at 48 h.

### Cell Invasion Assay

The cell invasion assay was performed using matrigel coated in Boyden chamber according to the manufacturer’s protocol (Cell Biolabs, CytoSelect ™ Cell Invasion Assay Kit). Mock and HCV-infected cells were serum starved, and approximately 1×10^6^ cells/ml was suspended in serum free media. Three hundred microliter of cell suspension was added onto the top of chamber and the lower chamber was filled with 500 µl DMEM media (10% FBS) and incubated at 37°C in 5% CO_2_. After 48 h, media was aspirated and non invasive cells were removed from top chamber using cotton swabs and stained with staining solution provided in the kit. Invasive cells in the bottom of the chamber were counted in high-power fields under an inverted microscope (Nikon, TE 2000-S, Japan), and extracted solutions were subjected to calorimetric analysis at 560 nm as per manufacturer’s instruction.

### Statistical Analysis

Error bars show the standard deviations of the means of data from three individual trials. Two-tailed unpaired *t*-tests were used to compare experimental conditions to those of the respective controls. In all test, *p*<0.05 was considered statistically significance.

## Results

### HCV Induces OPN Expression and Secretion

To determine the kinetics of OPN activation in HCV-infected cells, cellular lysates from mock (Huh7.5) and HCV-infected cells at various time points were subjected to western blot analysis. We observed significantly increased expression of precursor form of OPN (∼75 kDa) at days 3 to 8 (Fig. 1A, lane 4–9) followed by its cleavage into various forms of OPN (∼55 kDa, ∼42 kDa, ∼36 kDa) in HCV-infected cells compared to mock-infected cells. Interestingly, significant cleavage of all three forms of OPN was observed at day 8 postinfection (Fig. 1A, lane 9). Previously, full length OPN has been shown to be cleaved into various forms [38].

**Figure 1:** HCV activates OPN expression and secretion. (A) Mock (Huh7.5) and HCV-infected cells at days 1 to 8 postinfection were harvested and equal amounts of cellular lysates were subjected to immunoblot analysis using anti-OPN antibody. HCV NS3 represents HCV infection and actin was used as protein loading control. (B) Huh7.5 cells were infected with HCV at M.O.I. of 1. The cell culture supernatants were collected from HCV-infected cells at days 1 to 7, and were incubated with naive Huh7.5 cells. At day 4 postinfection, equal amount of cellular lysates were subjected to western blot analysis using anti-NS5A antibody. (C) Mock and HCV-infected cells at day 8 postinfection were incubated in serum free media overnight. Equal amounts of cell culture supernatants were subjected to western blot analysis using anti-OPN antibody. Immunoblot with anti-albumin was used as protein loading control. (D) HCV induces OPN mRNA expression. Total cellular RNA was extracted from mock and HCV-infected cells (day 8) followed by quantitative RT-PCR using OPN-specific primers. OPN gene expression was normalized by 18S rRNA. The values represent the means+SD of three independent experiments performed in duplicate. *denotes p<0.05 compared to mock cells (Huh7.5). (E) Equal amounts of cellular RNA from mock and HCV-infected cells as describe in panel D, were subjected to northern blot analysis using OPN probe. 28S rRNA probe was used as internal control.

To assess the cytotoxic effect of HCV-infected cells, mock and HCV-infected cells at days 2 to 8 postinfection were subjected to cell viability assay (Promega, Madison WI). The number of viable cells or metabolically active cells were observed using cell culture based quantitation of ATP. The results showed no significant cytotoxic effect by HCV-infection at days 2, 4, 6 and 8 postinfection (Fig. S1).

To determine the kinetics of HCV secretion from HCV-infected cells, Huh7.5 cells were incubated with HCV cell culture supernatants collected at various time points. The results show efficient secretion of HCV at day 4 to 7 (Fig. 1B).

To determine whether HCV infection induces secretion of OPN, cell culture supernatants from mock and HCV-infected Huh7.5 cells at day 8 postinfection were subjected to western blot analysis. We observed increased secretion of OPN (∼55 kDa, ∼42 kDa and ∼36 kDa) from HCV-infected cells compared to mock-infected cells (Fig. 1C, lane 2), suggesting that at later time point (day 8) HCV has the ability to process and secrete almost all forms of OPN.

To determine if the induction of OPN was due to increased expression of OPN mRNA, total cellular RNA was extracted from mock and HCV-infected cells (day 8) and OPN mRNA expression was quantified by RT-PCR. The results showed significantly higher OPN mRNA expression (∼5.5 fold) in HCV-infected cells compared to mock-infected cells (Fig. 1D). We also showed that HCV-infected cells expressed only full-length OPN mRNA (Fig. S2). To ascertain the presence of OPN mRNA in HCV-infected cells, OPN mRNA was partially sequenced and analysis was confirmed by comparing with the published nucleotide identity of human OPN gene. OPN partial amino acid sequences of Huh7.5 and HCV-infected cells with respect to known human OPN showed 100% identity (Fig. S3). To further characterize OPN mRNA, we performed northern blot analysis using OPN probe. We observed increased expression of full-length OPN mRNA in HCV-infected cells (Fig. 1E, lane 2), but no splice variants were observed. Taken together, these results suggest that HCV-infection stimulates synthesis, cleavage as well as secretion of OPN.

### Role of HCV-induced OPN on the Expression of Cell Surface Receptors, Integrin αVβ3 and CD44

To assess the level of infection, HCV-infected cells were immunostained using anti-NS5A antibody. The immunofluorescence microscopy results show more than 95% cells were infected by HCV (Fig. 2A). The above HCV-infected cells were transfected with siOPN and siGFP (control siRNA). Total cellular RNA was extracted and OPN mRNA expression was analyzed by QRT-PCR. The results showed increase OPN mRNA expression in HCV-infected cells which was reduced 15 fold (>90%) in HCV-infected cells transfected with siOPN but not with siGFP (Fig. 2B). Further to determine if HCV infection or HCV-induced OPN has any effect on αVβ3 and CD44 protein expression, equal amounts of cellular lysates from the cells transfected with above siRNA were subjected to western blot analysis. The results show no change in the expression of β3 or CD44 in HCV-infected cells or HCV-infected cells trasnfected with siOPN (Fig. 2C, D). In addition, we did not observe the expression of integrin β6, a negative control (Fig. 2C).

**Figure 2:** Effect of HCV-induced OPN on αVβ3 and CD44 expression. (A) Huh7.5 cells were incubated with HCV (m.o.i. of 1). At day 3 postinfection, cells were immunostained using anti-NS5A antibody as described in Materials and Methods. (B) Silencing of OPN mRNA expression. The above HCV-infected cells (panel A) were transfected with siGFP and siOPN using lipofectamine 2000 as per manufacturer’s instruction (Invitrogen). At 72 h posttransfection, cellular RNA was extracted and expression of OPN mRNA was quantified by QRT-PCR. OPN mRNA expression was normalized by 18S rRNA. Data represent means+standard deviations of two independent experiments performed in duplicate. *denotes p<0.05 compared to mock-infected Huh7.5 cells. **denotes p<0.05 compared to HCV-infected Huh7.5 cells transfected with siGFP. (C, D) Cellular lysates from the above siRNA transfected cells (panel B) were immunoblotted using anti-β3, anti-β6 and anti-CD44 antibodies. Actin was used as protein loading controls.

### HCV Induces Interaction of OPN with Cell Surface Receptors, Integrin αVβ3 and CD44

To determine the interaction of secreted OPN with integrin αVβ3 as well as CD44 at the cell surface, HCV-infected cells were transfected with siGFP or siOPN and were immunostained with antibodies against OPN, integrin αVβ3, CD44 and NS5A. The results showed colocalization of OPN with integrin αVβ3 as well as CD44 at the boundaries of HCV-infected cells compared to mock-infected cells (Fig. 3A, B). However, the colocalization was abrogated in HCV-infected cells transfected with siOPN but not with siGFP (control siRNA) (Fig. 3A, B). Taken together, these results indicate that the interaction of OPN with αVβ3 and CD44 occurs due to secretion of OPN from HCV-infected cells.

**Figure 3:** Colocalization of OPN with integrin αVβ3 and CD44. (A, B) Mock and HCV-infected cells (from figure 2A) were transfected with siGFP and siOPN. At 72 h posttransfection, cells were permeabilized and incubated with anti-OPN, anti-αVβ3, anti-CD44 and anti-HCV NS5A antibodies for 1 h at RT, followed by incubation with secondary antibodies; for OPN (anti-goat Alexa Fluor 546), αVβ3 (anti-mouse Alexa Fluor 488), CD44 (anti-mouse Alexa Fluor 488) and HCV NS5A (anti-rabbit Alexa Fluor 633). DAPI was used as a nuclear stain. Arrows represent colocalization of OPN with αVβ3 and CD44 respectively. HCV NS5A represents HCV infection. Scale bar 10 µM. (C) Colocalization of OPN with pan-cadherin (plasma membrane marker). Mock and HCV-infected cells (from figure 2A) were permeabilized and incubated with anti-OPN, anti-pan-cadherin and anti-HCV NS5A antibodies for 1 h at RT, followed by incubation with secondary antibodies; for OPN (anti-goat Alexa Fluor 546), pan-cadherin (anti-rabbit Alexa Fluor 488) and HCV NS5A (anti-rabbit Alexa Fluor 633). (D) Similarly, non-permeabilized mock and HCV-infected cells were incubated with anti-OPN and anti-pan-cadherin antibodies for 1 h at RT and then cells were permeabilized and incubated with anti-HCV NS5A antibody for 1 h at RT followed by 1 h incubation with above secondary antibodies. DAPI was used as a nuclear stain. Arrows represent colocalization of OPN with pan-cadherin. (E) Colocalization of OPN with PDI (ER marker). As described in panel C and D, permeabilized cells were incubated with anti-OPN, anti-PDI and anti-HCV NS5A antibodies for 1 h at RT, followed by incubation with secondary antibodies; for OPN (anti-goat Alexa Fluor 546), PDI (anti-rabbit Alexa Fluor 488) and HCV NS5A (anti-rabbit Alexa Fluor 633). (F) Simultaneously, non-permeabilized cells were incubated with anti-OPN and anti-PDI antibodies for 1 h at RT and then cells were permeabilized and incubated with anti-HCV NS5A antibody for 1 h at RT followed by 1 h incubation with above secondary antibodies. DAPI was used as a nuclear stain. Arrows represent colocalization of OPN with ER marker. HCV NS5A represents HCV infection. Scale bar 10 µM.

To verify the interaction of OPN with cell surface receptors (αVβ3 and CD44), mock (Huh7.5) and HCV-infected cells (permeabilized and nonpermeabilized) were immunostained with anti-pan-cadherin (plasma membrane marker), and anti-PDI (endoplasmic reticulum (ER) marker). The results show significant colocalization of OPN with pan-cadherin in permeabilized (Fig. 3C) and nonpermeabilized HCV-infected cells (Fig. 3D). However, few colocalization of OPN with ER marker was also observed only in permeabilized HCV-infected cells (Fig. 3E) but not in nonpermeabilized cells (Fig. 3F). These results suggest that secreted OPN interacts with cell surface receptors, integrin αVβ3 and CD44.

To determine the specificity of OPN interaction with integrin αVβ3 and CD44, HCV-infected cells were transfected with siOPN and siGFP. At 72 h postinfection, equal amounts of cellular lysates were immunoprecipitated using anti-OPN and immunoblotted with anti-β3 and anti-CD44. The results showed that OPN was able to pull down αVβ3 and CD44 in HCV-infected cells, which was abrogated in HCV-infected cells transfected with siOPN (Fig. 4, lane 4) but not with siGFP (Fig. 4, lane 3). In contrast, the immunoprecipitation using isotype control goat IgG antibody did not pull down αVβ3 and CD44 in HCV-infected cells (Fig. 4, lane 6, 8).

**Figure 4:** Interaction of OPN with integrin αVβ3 and CD44. HCV-infected Huh7.5 cells were transfected with siGFP and siOPN as described in Materials and Methods. At 72 h posttransfection, equal amounts of cellular lysates from mock, HCV-infected cells and HCV-infected cells transfected with above siRNA were immunoprecipitated using anti-OPN (1∶100) antibody and immunoblotted with anti-integrin β3 and anti-CD44 (lane 1–4). Similarly the cellular lysates from HCV-infected cells were immunoprecipitated with anti-OPN and isotype control goat IgG antibodies in two different sets followed by immunoblot analysis using anti-β3 and anti-CD44 (lane 5–8).

### HCV Induces EMT via OPN

To determine if activation of OPN in HCV-infected cells induces EMT, HCV-infected cells were transfected with siGFP or siOPN as described in figure 2B. Equal amounts of cellular lysates were immunoblotted with anti-E-cadherin (epithelial marker), anti-N-cadherin (mesenchymal marker), and anti-OPN. The results showed decreased expression of E-cadherin in HCV-infected cells compared to mock-infected cells (Fig. 5A, lane 2), which reappeared in HCV-infected cells transfected with siOPN (lane 4) but not with siGFP (lane 3). However, the expression of N-cadherin was increased in HCV-infected cells compared to mock-infected cells (Fig. 5B, lane 2), which was abrogated in cells transfected with siOPN (Fig. 5B, lane 4), but not with siGFP (lane 3). After siOPN transfection, we observed significant knock down of OPN expression (89% and 62%) in HCV-infected cells transfected with siOPN (Fig. 5A, B).

**Figure 5:** HCV induces EMT via OPN. HCV-infected cells were transfected with siOPN and siGFP as described in Materials and Methods. At 72 h posttransfection, cells were harvested and equal amounts of cellular lysates were immunoblotted with anti-E-cadherin (A), anti-N-cadherin (B), and anti-OPN (A, B). Actin was used as protein loading control.

### HCV-induced OPN Signaling Cascade

OPN is known to induce biological effects through signaling cascade by binding to cell surface receptors, integrin αVβ3 and CD44 [19]. To determine the role of HCV-induced OPN and its binding to αVβ3 and CD44 leading to signal transduction pathway, HCV-infected cells were transfected with siGFP, siOPN, siCD44, and siβ3. To demonstrate the effect of these siRNAs on the expression of their target genes, cellular lysates were subjected to western blot analysis using anti-OPN, anti-β3 and anti-CD44. The results showed significant reduction in the expression of OPN (∼69%), β3 (∼60%) and CD44 (∼67%) (Fig. 6A). These cellular lysates were immunoblotted using anti-FAK, anti-p-Src, and anti-p-Akt, the known players involved in integrin-mediated signaling pathways [19]. We observed increased phosphorylation/activation of FAK, Src, and Akt in HCV-infected cells which were reduced in cells transfected with siOPN, siCD44, and siβ3, but not with siGFP (Fig. 6B). Furthermore, our results showed that siβ3 was more effective in reducing the phosphorylation/activation of FAK, Src, and Akt compared to siCD44, indicating that CD44-mediated OPN signaling was less efficient compared to αVβ3 (Fig. 6B). In addition, we also observed reduced expression of N-cadherin in HCV-infected cells transfected with siOPN, siCD44 and siβ3, but not with siGFP (Fig. 6B). To validate that Huh7.5 cells induce above signaling pathway through the interaction of OPN at the cell surface receptors, mock (Huh7.5) cells were incubated with recombinant human OPN (rhOPN from R&D Systems) (50 nM) as described earlier [39]. The immunoblot results showed the increased phosphorylation/activation of FAK, Akt, N-cadherin and Src but decreased expression of E-cadherin in presence of rhOPN by western blot analysis (Fig. 6C, lane 2, 4).

**Figure 6:** Role of HCV-induced OPN in cell signaling cascade. (A) HCV-infected cells were transfected with siGFP, siOPN, siCD44, and siβ3 as described in Materials and Methods. At 72 h posttransfection, cells were harvested and equal amount of cellular lysates were subjected to western blot analysis using anti-OPN, anti-β3 and anti-CD44. (B) The above cellular lysates were subjected to western blot analysis using anti-FAK, anti-p-Akt (Ser ^473^), anti-p-Src (Tyr ^416^), and anti-N-cadherin antibodies. HCV NS3 was used as a representative of HCV-infection. (C) Mock (Huh7.5) cells were treated with recombinant human OPN (rhOPN) (50 nM) for 48 h. Cells were harvested and equal amounts of cellular lysates were immunoblotted using anti-FAK and anti-p-Akt (Ser^473^) (lane 1, 2), anti-E-cadherin, anti-N-cadherin, anti-pSrc ^416^ (lane 3, 4). (D) Cellular lysates from HepG2 cells incubated with cell culture supernatants from mock, HCV-infected cells and those infected cells transfected with siOPN and siGFP were immunoblotted using anti-E-cadherin and anti-N-cadherin (lane 1–4). Similarly cellular lysates from HepG2 cells incubated with cell culture supernatants from mock and HCV-infected cells with/without immunodepletion by anti-OPN, were immunoblotted using anti-E-cadherin and anti-N-cadherin (lane 5–7). Immunodepletion by isotype control goat IgG antibody was used as control (lane 8). Actin was used as protein loading control. The results shown are the representative of three independent experiments.

To demonstrate that the secretion of OPN from HCV-infected cells can induce paracrine cell signaling cascade and EMT, human hepatoblastoma cell line (HepG2) was incubated with cell culture supernatants from mock, HCV-infected cells and HCV-infected cells transfected with siGFP and siOPN. The results showed decreased expression of E-cadherin in HepG2 cells incubated with cell culture supernatant collected from HCV-infected cells (Fig. 6D, lane 2), which reappeared in HepG2 cells incubated with cell culture supernatant collected from HCV-infected cells transfected with siOPN (lane 4) but not with siGFP (lane 3). In contrast, the expression of N-cadherin was increased in HepG2 cells incubated with cell culture supernatant collected from HCV-infected cells (Fig. 6D, lane 2), that was abrogated in presence of cell culture supernatant collected from HCV-infected cells transfected with siOPN (Fig. 6D, lane 4), but not with siGFP (lane 3).

To further demonstrate the role of secreted OPN by HCV-infected Huh7.5 cells in EMT, OPN immunodepleted supernatant using anti-OPN antibody was incubated with HepG2 cells. The results show the increased expression of E-cadherin and decreased expression of N-cadherin in cells incubated with OPN immunodepleted supernatant (Fig. 6D, lane 7), which corresponds to HCV-infected cells transfected with siOPN (Fig. 6D, lane 4). In contrast, OPN immunodepleted supernatant using isotype control goat IgG did not show any effect (Fig. 6D, lane 8) similar to siGFP (Fig. 6D, lane 3). These results suggest that the secretion of OPN from HCV-infected cells was responsible for EMT in HepG2 cells.

### HCV-induces Hepatoma Cells Migration

To determine if HCV-induced OPN plays key role in human hepatoma cell migration, HCV-infected cells (from same pool of figure 2A) were transfected with siGFP and siOPN and were subjected to wound healing assay. The results showed increased cell migration in HCV-infected cells at 48 h post wounding which were reduced in HCV-infected cells transfected with siOPN, but not with siGFP (Fig. 7A). The increased migration depth at 48 h was recorded as ∼74% in HCV-infected cells which was reduced to ∼34% in HCV-infected cells transfected with siOPN (Fig. 7B), but not with siGFP (75%), suggesting the role of HCV-induced OPN in wound healing.

**Figure 7:** HCV induces hepatoma cells migration. (A) HCV-infected cells (from the same pool of figure 2A) were transfected with siGFP and siOPN and migration was examined by wound healing assay. Images were taken at 0 h and 48 h postwounding. Arrows indicate the wound of monolayer cells scratched using pipette tips. The results shown are representative of three independent experiments. (B) The percent migrated depth of above cells was measured in three independent experiments represented by bar diagram. *denotes p<0.05 compared to mock-infected Huh7.5 cells. **denotes p<0.05 compared to HCV-infected cells transfected with siGFP.

### HCV-induces Invasion of Hepatoma Cells

To demonstrate if OPN in HCV-infected cells induces cell invasion, HCV-infected cells (from same pool of figure 2A) were transfected with siGFP or siOPN and were placed in Boyden chamber (insert) coated with matrigel. The results showed the percent of HCV-infected cells invaded through the matrigel were recorded as ∼96% compared to mock cells (∼40%), which were significantly reduced ∼47% in HCV-infected cells transfected with siOPN, but not with siGFP (∼95%) (Fig. 8A, B).

**Figure 8:** HCV promotes invasion of hepatoma cells. (A) HCV-infected cells (from the same pool of figure 2A) were transfected with siGFP and siOPN. At 24 h posttransfection, approximately 3×10^5^ cells were seeded in transwell chamber for 48 h and images of invaded cells were recorded under microscope at least three individual fields per well at 10× magnification. (B) The invaded cells were counted in at least three individual fields per insert and represented by bar diagrams. The results shown are representative of two independent experiments performed in duplicate. (C) The above invaded cells were quantified in 96 wells plate at OD 560 nm using extraction buffer. Data represent means ± SD of two independent experiments performed in duplicate. *denotes p<0.05 compared to mock-infected Huh7.5 cells. **denotes p<0.05 compared to HCV-infected cells transfected with siGFP.

To further confirm these results, the invaded cells at the bottom of the inserts were extracted using extraction buffer and the absorbance was recorded at 560 nm. We observed ∼2.5 fold more invaded cells in HCV-infected cells which were reduced in siOPN transfected cells but not with siGFP, suggesting the role of HCV-induced OPN in hepatoma cell invasion (Fig. 8C).

### Activation of OPN in Primary Human Hepatocytes Infected with HCV

To examine if HCV-infection in primary human hepatocytes (PHH) activates OPN and induces OPN-mediated cell signaling cascade, cellular lysates from mock and HCV-infected hepatocytes were immunoblotted using anti-OPN, anti-β3, anti-CD44, anti-N-cadherin, anti-E-cadherin, anti-FAK, and anti-p-Akt. The results showed induction of precursor (∼75 kDa) and cleavage of precursor form into various forms (∼55, ∼42, ∼36 kDa) of OPN in HCV-infected primary human hepatocytes at day 8 postinfection (Fig. 9A). Our results also showed the equal expression of receptors, αVβ3 and CD44 in mock and HCV-infected primary hepatocytes (Fig. 9A), which is similar to what we observed in HCV-infected Huh7.5 cells (Fig. 2C, D). In addition, we also observed reduced expression of E-cadherin and increased expression of N-cadherin expression in HCV-infected primary human hepatocytes suggesting that HCV-induced EMT in primary human hepatocytes (Fig. 9B). Next we also observed increased phosphorylation/activation of FAK and Akt, involved in cell signaling cascade resulting in primary hepatocytes migration and invasion (Fig. 9B). To determine the level of HCV-infection, PHH and HCV-infected PHH were immunostained using anti-HCV NS5A antibody. The results showed about 75% of the cells were infected with HCV as observed by immunofluorescence microscopy (Fig. 9C). Taken together, these results validate our observation in HCV-infected human hepatoma cells.

**Figure 9:** HCV induces OPN and signaling cascade in primary human hepatocytes (PHH). (A, B) Equal amounts of cellular lysates from PHH (lane 1) and HCV-infected PHH (lane 2) were subjected to western blot analysis using anti-OPN, anti-CD44, anti-β3, anti-E-cadherin, anti-N-cadherin, anti-FAK, and anti-pAkt (Ser ^473^). HCV NS3 represents HCV infection and actin was used as protein loading control. (C) Immunofluorescence microscopy of HCV-infected PHH. HCV-infected PHH was incubated with HCV NS5A antibody for 1 h at RT followed by 1 h incubation with secondary HCV NS5A antibody (anti-rabbit Alexa Fluor 546) as describe in Materials and Methods. The magenta color indicates expression of HCV NS5A around the nucleus. Arrow indicates few uninfected cells. DAPI was used as a nuclear stain in blue color. Scale bar 10 µM. The results shown are the representative of three independent experiments.

## Discussion

HCC is one of the most common malignant tumors which has a very high mortality rate due to its high incidence of invasion and metastasis [5], [6]. It is a complex and heterogeneous tumor with a multistep process involving multiple cellular signaling pathways [40]. HCV induces chronic liver injury that can lead to progressive fibrosis, cirrhosis and is one of the leading causes of HCC [40]. HCV-associated HCC has been reported to be associated with an increased recurrence after liver resection suggesting that HCV may promote tumor growth and metastasis [41]. However, the underlying mechanisms responsible for invasiveness and metastatic spread of HCV-induced HCC are still not fully understood. Previous studies have indicated that OPN is involved in tumor metastasis and has been detected in numerous cancers including HCC, suggesting a correlation between high levels of OPN expression and malignant invasion [21], [23]. Studies have also shown higher levels of OPN during liver injury, inflammation as well as in the plasma of HCV related HCC patients than in healthy individuals [42]–[46]. Recent studies have identified OPN as a novel marker for early diagnosis of HCC [47]. However, the role of OPN in HCV-induced HCC is not known.

In this study, we determined the induction of OPN and then investigated the interaction of secreted OPN with cell surface receptors, integrin αVβ3 and CD44 leading to EMT, migration and invasion of human hepatocytes. Full-length OPN is composed of about 314 amino acids and there are also functionally important cleaved products and occasional splice variants [24], [38], [48]. In HCV-infected hepatoma cells, we could observe only full-length OPN mRNA (Fig. S2 and Fig. 1E), indicating that HCV-infection does not induce the formation of OPN splice variants. In contrast, recent studies have shown the formation of two splice variants of OPN in HCC [48]. This could be due to different cell types and the source of HCC tissue samples used in those studies. The molecular weight of OPN varies from ∼44 to ∼75 kDa because of altered glycosylation and phosphorylation [49], [50]. In this study, we observed full-length OPN polypeptide (∼75 kDa), which is cleaved in HCV-infected cells as well as in primary human hepatocytes (Fig. 1A and 9A) and secreted as ∼55 kDa, ∼42 kDa and ∼36 kDa OPN (Fig. 1C). However, the underlying mechanisms by which HCV-induced the proteolytic processing of OPN is not known. These results are consistent with the previous reports indicating that OPN acts as a novel substrate for thrombin, matrix metalloproteases (MMPs), and the cleaved fragments enhanced adhesion and migration *in vitro* through ligation to receptors including integrins [19], [51]–[53]. All the secreted forms of OPN from HCV-infected cells may bind with cell surface receptors and induce signaling cascade.

OPN exists both as a component of the extracellular matrix and a secreted multifunctional cytokine [30], [31]. Previous studies have shown that OPN binds to the family of αVβ integrins, and the cell surface adhesion molecule CD44, to initiate cellular signals that enable tumor progression [19], [54]. The interaction of OPN with integrins is dependent on the OPN Arg-Gly-Asp (RGD) motif and on a high activation state of the integrin receptors, αVβ1, αVβ3 and αVβ5 [55]. The widely expressed αVβ3-integrin is a well characterized receptor of OPN in processes such as cell adhesion, migration, and bone resorption [19], [56]. The C-terminal region of OPN binds to CD44 to induce cellular signal responsible for tumor progression [57]. Based on these reports we focused on determining the interaction of αVβ3 and CD44 with OPN. Our results showed colocalization of OPN with αVβ3 and CD44 at the surface of HCV-infected cells, suggesting the binding of secreted OPN to αVβ3 integrin as well as CD44 receptors (Fig. 3A, B), which can signals through various signaling cascade events leading to metastasis of HCV-infected hepatocyes. These results are consistent with the previous report, where the interaction of secreted OPN with cellular receptors such as integrins and CD44 are more efficient than native OPN, and associated with cell migration, invasion and metastasis of a number of malignant tumours, including HCC [19], [23], [38].

Previously, it has been shown that the binding of OPN to integrin β1 and β3 receptors leads to phosphorylation of FAK and Src, which in turn initiate signals for proliferation, cytoskeletal organization, and motility [32], [58]. OPN can also bind to CD44 and acts as a signaling molecule to participate in series of related molecular processes, such as adhesion, cell migration and signal transduction [49], [59], [60]. Moreover, OPN function *in vivo* is multifaceted, tissue specific, and involves multiple signaling pathways that are mediated by the αVβ3 integrin and CD44 receptors during the step-wise progression of metastasis [38], [61]. A well known member of the non-receptor protein tyrosine kinase family, c-Src, plays a crucial role in signaling downstream of integrin receptors [62]. In addition, its association with several focal-adhesion proteins such as FAK, paxillin and vinculin also regulates cell attachment, spreading, and remodeling and turnover of focal adhesions [63]. Some known downstream effectors of OPN include PI3-kinase/Akt, NF-kB, and MMPs have been shown to mediate critical metastatic processes such as ECM (extra cellular matrix) proteolysis, remodeling, and cell migration [24], [64]. In our finding, interaction of OPN with integrin αVβ3 and CD44 induced phosphorylation/activation of FAK, Akt, Src and induction of N-cadherin leading to EMT, cell migration and invasion in HCV-infected hepatoma cells as well as in primary human heptocytes (Fig. 6 B, C and Fig. 9B), which are consistent to the previous reports where HCV infection or HCV proteins have been shown to play critical role in EMT and metastasis [65], [66].

E-cadherin, is a transmembrane glycoprotein that is primarily expressed in epithelia at the sites of cell-cell contacts. In most cancers of epithelial origin, E-cadherin-mediated cell-cell adhesion is lost concomitantly with progression toward tumor malignancy [67]. Loss of E-cadherin promotes the progression from adenoma to carcinoma. Our results show the loss of E-cadherin expression, and gain of N-cadherin expression which was dependent on HCV-induced OPN in human hepatocytes. In addition, we also observed OPN dependent loss and gain of E-cadherin and N-cadherin expression, respectively, suggesting the paracrine effect of OPN on HepG2 cell line (Fig. 6D), which is consistent to the growth of Huh7, HepG2 and HeLa cells in the presence of OPN conditioned media [48]. In normal physiological conditions, OPN plays a key role in cell migration [68]. Our findings suggest that HCV has the ability to promote migration (Fig. 7) and invasion (Fig. 8) of hepatocytes via induction and secretion of OPN. These results are consistent with the previous reports on the role of HCV infection and the expression of HCV NS5A and E/E2 in EMT and the migration of hepatocytes [65], [66], [69].

In summary, our results provide for the first time clear evidence demonstrating the induction and secretion of OPN from HCV-infected hepatocytes. The secreted OPN induces EMT and metastasis via binding to cell surface receptor αVβ3 and CD44 (Fig. 10). Silencing of OPN expression by OPN siRNA and immunodepletion of OPN by anti-OPN antibody resulted in reduced EMT, migration, and invasion of human hepatocytes, which may be a useful target in developing a better therapeutic strategy for liver cancer associated with chronic hepatitis C. Our results also provide novel insight into the mechanisms of HCV-infected hepatocytes migration and HCC.

**Figure 10:** Model illustrating the OPN mediated signaling cascade in HCV-infected hepatocytes. HCV induces OPN expression, which is cleaved by unknown mechanism in response to HCV-infection and the active forms are secreted out from the cells. The secreted form of OPN binds to cell surface receptors on the same or other cells via integrin αVβ3 and CD44. This interaction leads to EMT, cell migration and invasion through the activation/phosphorylation of FAK, Akt and Src mediated signaling pathways.

## Supporting Information

Figure S1 Cell Viability of HCV infected Huh7.5 cells. Mock (Huh7.5) and HCV-infected cells at various time points were placed in 96 wells plate. The cells were lysed and ATP was quantitated as per manufacturer’s instruction using CellTitre-Glo Luminescent Cell viability Assay Kit (Promega). The percent viability was calculated considering 100% viability for mock cells compare to HCV-infected cells. We observed 98.8%, 113%, 110% and 94.7% cell viability of HCV-infected cells at day 2, 4, 6 and 8 postinfection respectively. The values represent the means ± SD of three independent experiments performed in duplicate.
(TIF)

Figure S2 HCV activates OPN mRNA expression. Mock and HCV-infected cells were harvested and total cellular RNA was extracted using TRIzol (Invitrogen) followed by cDNA synthesis. OPN mRNA was amplified using OPN-specific primers by semi-quantitative RT-PCR. The equal volume of PCR products were loaded onto 1% agarose gel. OPN gene expression was compared by 18S rRNA. We observed single OPN band which correspond to the size of full length OPN.
(TIF)

Figure S3 Alignment of deduced partial amino acid sequences of OPN protein. Total RNA was extracted by TRIzol (Invitrogen, CA) from mock (Huh7.5) and HCV-infected cells and cDNA was transcribed and amplified by conventional PCR using GoTaq® Green master mix kit (Promega Corporation, Madison, Wisconsin,USA) using OPN specific primers (described in Materials and Methods). Amplified OPN PCR products were verified on 1% agarose gel electrophoresis and the remaining amplified products were subjected to column purification using QIAquick PCR Puirfication Kit (Qiagen, GmbH, Hilden, Germany). Purified PCR products were partially sequenced by dideoxynucleotides chain termination method (Fredrick Sanger) in automated ABI 3730 High-Throughput DNA Sequencer (Applied Biosystem, Foster City, USA) at the Genomics Core facility of Center for Genetic Medicine in Northwestern University (Chicago, IL, USA). Resultant sequences were compared with published cognate sequences of corresponding genes by BLAST and the amino acid (aa) sequences were deduced by the DNA sequence translation tool EMBOSS-Transeq (EMBL-EBI Group). Alignment of the deduced partial amino acid sequences of OPN protein of mock and HCV-infected Huh7.5 cells with respect to published human OPN protein sequence was carried out using Clustal W2 software. The OPN sequences of Huh7.5, HCV-infected Huh7.5 cells, and reference human OPN were indicated as ‘Osteopontin Huh7.5′, ‘Osteopontin HCV’ and ‘Osteopontin (*Homo sapiens*)’, respectively.
(TIF)

## References

[1] Di Bisceglie AM (1997) Hepatitis C and hepatocellular carcinoma. Hepatology 26 (Suppl): S34–S38.10.1002/hep.5102607069305661

[2] BlightKJ, KolykhalovAA, RiceCM (2000) Efficient initiation of HCV RNA replication in cell culture. Science 290: 1972–1974.11110665 10.1126/science.290.5498.1972

[3] WakitaT, PietschmannT, KatoT, DateT, MiyamotoM, et al. (2005) Production of infectious hepatitis C virus in tissue culture from a cloned viral genome. Nat Med 11: 791–796.15951748 10.1038/nm1268PMC2918402

[4] ZhongJ, GastaminzaP, ChengG, KapadiaS, KatoT, et al. (2005) Robust hepatitis C virus infection in vitro. Proc Natl Acad Sci 102: 9294–9299.15939869 10.1073/pnas.0503596102PMC1166622

[5] ParkinDM, BrayF, FerlayJ, PisaniP (2002) Global cancer statistics. CA Cancer J Clin 55: 74–108.10.3322/canjclin.55.2.7415761078

[6] LlovetJM, BruixJ (2008) Molecular targeted therapies in hepatocellular carcinoma. Hepatology 48: 1312–1327.18821591 10.1002/hep.22506PMC2597642

[7] Di BisceglieAM, LyraAC, SchwartzM, ReddyRK, MartinP, et al. (2003) Hepatitis C-related hepatocellular carcinoma in the United States: influence of ethnic status. Am J Gastroenterol 98: 2060–2063.14499788 10.1111/j.1572-0241.2003.t01-1-07641.x

[8] ChenXP, QiuFZ, WuZD, ZhangZW, HuangZY, et al. (2006) Long-term outcome of resection of large hepatocellular carcinoma. Br J Surg 93: 600–606.16607679 10.1002/bjs.5335

[9] KernMA, BreuhahnK, SchirmacherP (2002) Molecular pathogenesis of human hepatocellular carcinoma. Adv Cancer Res 86: 67–112.12374281 10.1016/s0065-230x(02)86003-1

[10] HassanM, GhozlanH, Abdel-KaderO (2005) Activation of c-Jun NH2-terminal kinase (JNK) signaling pathway is essential for the stimulation of hepatitis C virus (HCV) non-structural protein 3 (NS3)-mediated cell growth. Virology 333: 324–336.15721365 10.1016/j.virol.2005.01.008

[11] KasprzakA, AdamekA, PrzybyszewskaW, OlejniczakK, BiczyskoW, et al. (2009) p21/Wafl/Cipl cellular expression in chronic long-lasting hepatitis C: correlation with HCV proteins (C, NS3, NS5A), other cell-cycle related proteins and selected clinical data. Folia Histochem Cytobiol 47: 385–394.20164022 10.2478/v10042-009-0096-x

[12] HeQQ, ChengRX, SunY, FengDY, ChenZC, et al. (2003) Hepatocyte transformation and tumor development induced by hepatitis C virus NS3 c-terminal deleted protein. World J Gastroenterol 9: 474–478.12632500 10.3748/wjg.v9.i3.474PMC4621564

[13] MoriyaK, FujieH, ShintaniY, YotsuyanagiH, TsutsumiT, et al. (1998) The core protein of hepatitis-C virus induces hepatocellular carcinoma in transgenic mice. Nat Med 4: 1065–1067.9734402 10.1038/2053

[14] MoradpourD, EnglertC, WakitaT, WandsJR (1996) Characterization of cell lines allowing tightly regulated expression of hepatitis-C virus core protein. Virology 222: 51–63.8806487 10.1006/viro.1996.0397

[15] MoriyaK, NakagawaK, SantaT, ShintaniY, FujieH, et al. (2001) Oxidative stress in the absence of inflammation in a mouse model for hepatitis C virus-associated hepatocarcinogenesis. Cancer Res 61: 4365–4370.11389061

[16] FarinatiF, CardinR, De MariaN, Della LiberaG, MarafinC, et al. (1995) Iron storage, lipid peroxidation and glutathione turnover in chronic anti-HCV positive hepatitis. J Hepatol 22: 449–456.7545199 10.1016/0168-8278(95)80108-1

[17] GongG, WarisG, TanveerR, SiddiquiA (2001) Human hepatitis C virus NS5A protein alters intracellular calcium levels, induces oxidative stress, and activates STAT-3 and NF-kappa B. Proc Natl Acad Sci. 98: 9599–9604.10.1073/pnas.171311298PMC5549811481452

[18] PresserLD, HaskettA, WarisG (2011) Hepatitis C virus-induced furin and thrombo-spondin-1 activate TGF-β1: role of TGF-β1 in HCV replication. Virology 412: 284–296.21296375 10.1016/j.virol.2010.12.051PMC3073624

[19] RangaswamiH, BulbuleA, KunduGC (2006) Osteopontin: role in cell signaling and cancer progression. Trends Cell Biol 16: 79–87.16406521 10.1016/j.tcb.2005.12.005

[20] PanHW, OuYH, PengSY, LiuSH, LaiPL, et al. (2003) Overexpression of osteopontin is associated with intrahepatic metastasis, early recurrence, and poorer prognosis of surgically resected hepatocellular carcinoma. Cancer 98: 119–127.12833464 10.1002/cncr.11487

[21] GotohM, SakamotoM, KanetakaK, ChuumaM, HirohashiS (2002) Overexpression of osteopontin in hepatocellular carcinoma. Pathology International 52: 19–24.11940202 10.1046/j.1440-1827.2002.01316.x

[22] SengerDR, WirthDF, HynesRO (1979) Transformed mammalian cells secrete specific proteins and phosphoproteins. Cell 16: 885–893.88265 10.1016/0092-8674(79)90103-x

[23] OatesAJ, BarracloughR, RudlandPS (1997) The role of osteopontin in tumorigenesis and metastasis. Invasion Metastasis 17: 1–15.9425320

[24] WaiPY, KuoPC (2008) Osteopontin: regulation in tumor metastasis. Cancer Metastasis Rev 27: 103–118.18049863 10.1007/s10555-007-9104-9

[25] PatourauxS, BonnafousS, VoicanCS, AntyR, Saint-PaulMC, et al. (2012) The osteopontin level in liver, adipose tissue and serum is correlated with fibrosis in patients with alcoholic liver disease. PLoS One 7: e35612 doi:10.1371/journal.pone.003561222530059 PMC3329460

[26] WhalenKA, WeberGF, BenjaminTL, SchaffhausenBS (2008) Polyomavirus middle T antigen induces the transcription of osteopontin, a gene important for the migration of transformed cells. J Virol 82: 4946–4954.18337582 10.1128/JVI.02650-07PMC2346735

[27] ZhangX, YeLH, ZhangXD (2010) A mutant of hepatitis B virus X protein (HBx Delta 127) enhances hepatoma cell migration via osteopontin involving 5-lipoxygenase. Acta Pharmacol Sin 31: 593–600.20364155 10.1038/aps.2010.36PMC4002751

[28] BrownA, IslamT, AdamsR, NerleS, KamaraM, et al. (2011) Osteopontin enhances HIV replication and is increased in the brain and cerebrospinal fluid of HIV-infected individuals. J Neurovirol 17: 382–392.21556958 10.1007/s13365-011-0035-4PMC3331788

[29] Iqbal J, McRae S, Banaudha K, Mai T, Waris G (2013) Mechanism of HCV-induced Osteopontin and its role in epithelial to mesenchymal transition of hepatocytes. J Biol Chem [Epub ahead of print].10.1074/jbc.M113.492314PMC387355724240095

[30] KazaneckiCC, UzwiakDJ, DenhardtDT (2007) Control of osteopontin signaling and function by post-translational phosphorylation and protein folding. J Cell Biochem 102: 912–924.17910028 10.1002/jcb.21558

[31] UedeT (2011) Osteopontin, intrinsic tissue regulator of intractable inflammatory diseases. Pathol Int 61: 265–280.21501293 10.1111/j.1440-1827.2011.02649.x

[32] WaiPY, CaoPC (2004) The role of Osteopontin in tumor metastasis. J Surg Res 121: 228–241.15501463 10.1016/j.jss.2004.03.028

[33] BlightKJ, McKeatingJA, RiceCM (2002) Highly permissive cell lines for subgenomic and genomic hepatitis C virus RNA replication. J Virol 76: 13001–14.12438626 10.1128/JVI.76.24.13001-13014.2002PMC136668

[34] RaneyAK, MilichDR, McLachlanA (1989) Characterization of hepatitis B virus major surface antigen gene transcriptional regulatory elements in differentiated hepatoma cell lines. J Virol 63: 3919–25.2548006 10.1128/jvi.63.9.3919-3925.1989PMC250988

[35] BurdetteD, HaskettA, PresserL, McRaeS, IqbalJ, et al. (2012) Hepatitis C virus activates interleukin-1β via caspase-1-inflammasome complex. J Gen Virol 93: 235–246.21994322 10.1099/vir.0.034033-0PMC3352344

[36] SchaeferB, Rivas-EstillaAM, Meraz-CruzN, Reyes-RomeroMA, Hernández-NazaraZH, et al. (2003) Reciprocal modulation of matrix metalloproteinase-13 and type I collagen genes in rat hepatic stellate cells. Am J Pathol 162: 1771–1780.12759235 10.1016/S0002-9440(10)64312-XPMC1868138

[37] BanaudhaK, OrensteinJM, KorolnekT, St LaurentGC3rd, WakitaT, et al. (2010) Primary hepatocyte culture supports hepatitis C virus replication: a model for infection- associated hepatocarcinogenesis. Hepatology 51: 1922–1932.20512986 10.1002/hep.23616

[38] SengerDR, LedbetterSR, ClaffeyKP, Papadopoulos-SergiouA, PeruzziCA, et al. (1996) Stimulation of endothelial cell migration by vascular permeability factor/vascular endothelial growth factor through cooperative mechanisms involving the alphavbeta3 integrin, osteopontin, and thrombin. Am J Pathol 149: 293–305.8686754 PMC1865227

[39] ZhangR, PanX, HuangZ, WeberGF, ZhangG (2011) Osteopontin enhances the expression and activity of MMP-2 via the SDF-1/CXCR4 axis in hepatocellular carcinoma cell lines. PLoS One 6: e23831 doi:10.1371/journal.pone.002383121909361 PMC3166084

[40] FaraziPA, DePinhoRA (2006) Hepatocellular carcinoma pathogenesis: from genes to environment. Nat Rev Cancer 6: 674–687.16929323 10.1038/nrc1934

[41] HuangYH, WuJC, ChenCH, ChangTT, LeePC, et al. (2005) Comparison of recurrence after hepatic resection in patients with hepatitis B vs. hepatitis C-related small hepatocellular carcinoma in hepatitis B virus endemic area. Liver Int 25: 236–241.15780044 10.1111/j.1478-3231.2005.01081.x

[42] De MinicisS, SekiE, UchinamiH, KluweJ, ZhangY, et al. (2007) Gene expression profiles during hepatic stellate cell activation in culture and in vivo. Gastroenterology 132: 1937–1946.17484886 10.1053/j.gastro.2007.02.033

[43] SynWK, ChoiSS, LiaskouE, KaracaGF, AgboolaKM, et al. (2011) Osteopontin is induced by hedgehog pathway activation and promotes fibrosis progression in nonalcoholic steatohepatitis. Hepatology 53: 106–115.20967826 10.1002/hep.23998PMC3025083

[44] LeeSH, SeoGS, ParkYN, YooTM, SohnDH (2004) Effects and regulation of osteopontin in rat hepatic stellate cells. Biochem Pharmacol 68: 2367–2378.15548383 10.1016/j.bcp.2004.08.022

[45] LorenaD, DarbyIA, GadeauAP, LeenLL, RittlingS, et al. (2006) Osteopontin expression in normal and fibrotic liver altered liver healing in osteopontin-deficient mice. J Hepatol 44: 383–390.16221502 10.1016/j.jhep.2005.07.024

[46] Abu El MakaremMA, Abdel-AleemA, AliA, SaberR, ShatatM, et al. (2011) Diagnostic significance of plasma osteopontin in hepatitis C virus-related hepatocellular carcinoma. Annals of Hepatology 10: 296–305.21677331

[47] ShangS, PlymothA, GeS, FengZ, RosenHR, et al. (2012) Identification of osteopontin as a novel marker for early hepatocellular carcinoma. Hepatology 55: 483–490.21953299 10.1002/hep.24703PMC3914762

[48] PhillipsRJ, HelbigKJ, Van der HoekKH, SethD, BeardMR (2012) Osteopontin increases hepatocellular carcinoma cell growth in a CD44 dependant manner. World J Gastroenterol 18: 3389–3399.22807608 10.3748/wjg.v18.i26.3389PMC3396191

[49] SodekJ, GanssB, Mc KeeMD (2000) Osteopontin. Critical Reviews in Oral Biology and Medicine 11: 279–303.11021631 10.1177/10454411000110030101

[50] PrinceCW, OosawaT, ButlerWT, TomanaM, BhownAS, et al. (1987) Isolation, characterization, and biosynthesis of a phosphorylated glycoprotein from rat bone. J Biol Chem 262: 2900–2907.3469201

[51] JohnsonGA, BurghardtRC, JoyceMM, SpencerTE, BazerFW, et al. (2003) Osteopontin is synthesized by uterine glands and a 45-kDa cleavage fragment is localized at the uterine-placental interface throughout ovine pregnancy. Biol Reprod 69: 92–98.12606367 10.1095/biolreprod.102.013573

[52] TakafujiV, ForguesM, UnsworthE, GoldsmithP, WangXW (2007) An osteopontin fragment is essential for tumor cell invasion in hepatocellular carcinoma. Oncogene 26: 6361–6371.17452979 10.1038/sj.onc.1210463

[53] KimHJ, LeeHJ, JunJI, OhY, ChoiSG, et al. (2009) Intracellular cleavage of osteopontin by caspase-8 modulates hypoxia/reoxygenation cell death through p53. Proc Natl Acad Sci 106: 15326–15331.19706414 10.1073/pnas.0903704106PMC2729277

[54] KikuchiS, GriffinCT, WangSS, BissellDM (2005) Role of CD44 in epithelial wound repair: migration of rat hepatic stellate cells utilizes hyaluronic acid and CD44v6. J Biol Chem 280: 15398–15404.15691832 10.1074/jbc.M414048200

[55] FurgerKA, AllanAL, WilsonSM, HotaC, VantyghemSA, et al. (2003) Beta (3) integrin expression increases breast carcinoma cell responsiveness to the malignancy-enhancing effects of osteopontin. Mol Cancer Res 1: 810–819.14517343

[56] ChristensenB, SchackL, KläningE, SørensenES (2010) Osteopontin is cleaved at multiple sites close to its integrin-binding motifs in milk and is a novel substrate for plasmin and cathepsin D. J Biol Chem. 285: 7929–7937.10.1074/jbc.M109.075010PMC283294320071328

[57] WeberGF, AshkarS, GlimcherMJ, CantorH (1996) Receptor-ligand interaction between CD44 and osteopontin (Eta-1). Science 271: 509–512.8560266 10.1126/science.271.5248.509

[58] ZouC, LuoQ, QinJ, ShiY, YangL, et al. (2013) Osteopontin Promotes Mesenchymal Stem Cell Migration and Lessens Cell Stiffness via Integrin β1, FAK, and ERK Pathways. Cell Biochem Biophys 65: 455–462.23086356 10.1007/s12013-012-9449-8

[59] WeberGF, CantorH (1996) The immunology of Eta-1/osteopontin. Cytokine Growth Factor Rev 7: 241–248.8971479 10.1016/s1359-6101(96)00030-5

[60] GeorgoliosA, BatistatouA, ManolopoulosL, CharalabopoulosK (2006) Role and expression patterns of E-cadherin in head and neck squamous cell carcinoma (HNSCC). J Exp Clin Cancer Res 25: 5–14.16761612

[61] GaoC, GuoH, WeiJ, KuoPC (2003) Osteopontin inhibits expression of cytochrome c oxidase in RAW 264.7 murine macrophages. Biochem Biophys Res Commun 309: 120–125.12943672 10.1016/s0006-291x(03)01534-1

[62] AlperO, BowdenET (2005) Novel insights into c-Src. Curr Pharm Des 11: 1119–1130.15853660 10.2174/1381612053507576

[63] VolbergT, RomerL, ZamirE, GeigerB (2001) pp60 (c-Src) and related tyrosine kinases: a role in the assembly and reorganization of matrix adhesion. J Cell Sci 114: 2279–2289.11493667 10.1242/jcs.114.12.2279

[64] NicholsonKM, AndersonNG (2002) The protein kinase B/Akt signalling pathway in human malignancy. Cell Signal 14: 381–395.11882383 10.1016/s0898-6568(01)00271-6

[65] BoseSK, MeyerK, Di BisceglieAM, RayRB, RayR (2012) Hepatitis C virus induces epithelial-mesenchymal transition in primary human hepatocytes. J Virol 86: 13621–13628.23035229 10.1128/JVI.02016-12PMC3503076

[66] AkkariL, GrégoireD, Floc’hN, MoreauM, HernandezC, et al. (2012) Hepatitis C viral protein NS5A induces EMT and participates in oncogenic transformation of primary hepatocyte precursors. J Hepatol 57: 1021–1028.22750466 10.1016/j.jhep.2012.06.027

[67] HirohashiS (1998) Inactivation of the E-cadherin-mediated cell adhesion system in human cancers. Am J Pathol 153: 333–339.9708792 10.1016/S0002-9440(10)65575-7PMC1852964

[68] LiuYN, KangBB, ChenJH (2004) Transcriptional regulation of human osteopontin promoter by C/EBPa and AML-1 in metastatic cancer cells. Oncogene 23: 278–288.14712233 10.1038/sj.onc.1207022

[69] WilsonGK, BrimacombeCL, RoweIA, ReynoldsGM, FletcherNF, et al. (2012) A dual role for hypoxia inducible factor-1α in the hepatitis C virus lifecycle and hepatoma migration. J Hepatol 56: 803–809.22178269 10.1016/j.jhep.2011.11.018PMC3343261

